# NR2F2-AS1 accelerates cell proliferation through regulating miR-4429/MBD1 axis in cervical cancer

**DOI:** 10.1042/BSR20194282

**Published:** 2020-06-15

**Authors:** Dan Liu, Kejin Huang, Tiaojiao Wang, Xufeng Zhang, Wentao Liu, Xiaolong Yue, Jin Wu

**Affiliations:** 1 The Seventh Department of the Internal Medicine, Harbin Medical University Cancer Hospital, Harbin 150081, Heilongjiang, China; 2 Department of Gynecology, Harbin Medical University Cancer Hospital, Harbin 150081, Heilongjiang, China

**Keywords:** cervical cancer, MBD1, miR-4429, NR2F2-AS1

## Abstract

Cervical cancer is one of the most frequent malignant tumors in female. Increasing studies have demonstrated that long noncoding RNAs (lncRNAs) play a key role in the development of multiple cancers. Although some studies have confirmed that lncRNA NR2F2 antisense RNA 1 (NR2F2-AS1) is a pro-cancer gene in many cancers, the molecular mechanism of NR2F2-AS1 in cervical cancer has not been completely elucidated. In the present study, our results revealed that NR2F2-AS1 expression was up-regulated in cervical cancer tissues and cells, notably in patients with advanced cervical cancer. NR2F2-AS1 accelerated progression of cervical cancer by facilitating cell proliferation, migration, invasion, and EMT process, but inhibiting cell apoptosis. Moreover, NR2F2-AS1 acted as a molecular sponge of miR-4429 and methyl-CpG-binding domain protein 1 (MBD1) was a downstream target of miR-4429 in cervical cancer. Furthermore, there was a negative correlation between miR-4429 expression and NR2F2-AS1 or MBD1 expression in tumor tissues. Rescue experiments confirmed that MBD1 overexpression partly rescued NR2F2-AS1 knockdown-mediated inhibition of progression in cervical cancer. To sum up, these results suggested the potential mechanism of NR2F2-AS1 in cervical cancer and revealed that NR2F2-AS1 exerted its carcinogenic effect via regulating miR-4429/MBD1 axis, indicating a promising insight into the therapeutic target of cervical cancer.

## Introduction

Cervical cancer is the second malignant tumor among women worldwide, with high morbidity and mortality every year. Almost 85% of cases occur in poor and developing countries [1,2]. High-risk HPV infection is the main cause of cervical cancer [3,4]. Although great strides have been made in the diagnostic methods and treatment strategies of cervical cancer, the overall survival rate of the patients remains unsatisfactory partially due to its late detection and recurrence [5,6]. Hence, it is of great necessity to illuminate the underlying molecular mechanisms of cervical cancer.

The long noncoding RNAs (lncRNAs) are a group of noncoding RNAs with more than 200 nucleotides that participate in many physiological and pathological processes of malignancies [7,8]. Mounting evidence has also suggested that lncRNAs were critical regulators in the progression of numerous cancers. For example, lncRNA TTN-AS1 promotes cell proliferation and invasion in colorectal cancer by absorbing miR-376a-3p to up-regulate KLF15 [9]. LncRNA LINC01314 inhibits cell migration, invasion and angiogenesis through modulating KLK4 in gastric cancer [10]. LncRNA LINC00052 accelerates the progression of head and neck squamous cell carcinoma via targeting miR-608/EGFR axis [11]. There is proof that as a member of lncRNAs, NR2F2 antisense RNA 1 (NR2F2-AS1) acts as a tumor promoter in some cancers. For instance, NR2F2-AS1 aggravates the progression of prostate carcinoma via CDK4 elevation [12]. NR2F2-AS1 sponges miR-320b to facilitate tumorigenesis through increasing BMI1 expression in non-small cell lung cancer [13]. Knockdown of NR2F2-AS1 causes G1 arrest of colorectal cancer cells via repressing CDK6 [14]. Nevertheless, the regulatory mechanism and biological function of NR2F2-AS1 in cervical cancer are obscure.

In the present study, we aimed to investigate the specific function and regulatory mechanism of NR2F2-AS1 in cervical cancer. Our results showed that NR2F2-AS1 accelerated cervical cancer progression through sponging miR-4429 to modulate methyl-CpG-binding domain protein 1 (MBD1), which may promote the development of therapeutic strategies of cervical cancer.

## Materials and methods

### Clinical samples

The cervical cancer tissues and noncancerous tissues were collected from patients with cervical cancer via surgical resection at Harbin Medical University Cancer Hospital (Heilongjiang, China). All samples were stored at −80°C. Before the operation, these patients received no other anticancer treatment. All informed consents were obtained from patients before surgery, and the present study was approved by the Ethics Committee of Harbin Medical University Cancer Hospital (Heilongjiang, China).

### Cell lines

Cervical cancer cell lines (HeLa, SiHa, C33A, and C4-1) and normal human cervical cells (Ect1/E6E7) were provided by the American Type Culture Collection (ATCC; Manassas, VA, U.S.A.). All cells were cultured in Dulbecco’s modified Eagle’s medium (DMEM) containing 10% fetal bovine serum (FBS). Cells were maintained in the humidified atmosphere with 5% CO_2_ at 37°C.

### Transfection

Sh-NR2F2-AS1#1 and sh-NR2F2-AS1#2 were transfected into HeLa and SiHa cells to knockdown NR2F2-AS1 and shNC was utilized as negative control. MBD1 was overexpressed with pcDNA3.1 vector, and miR-4429 was overexpressed with miR-4429 mimics. Plasmids transfections were conducted by Lipofectamine 2000 (Invitrogen, Carlsbad, CA, U.S.A.) in accordance with the manufacturer’s protocol. Cells were incubated for 24 h after transfection and then were purified for the next experiments. These synthesized plasmids were all purchased from GenePharma (Shanghai, China).

### RNA extraction and quantitative real-time PCR

Total RNA was extracted from HeLa or SiHa cells with Trizol reagent (Takara, Otsu, Japan). Extracted RNA was reverse transcribed into complementary DNA (cDNA) (Amersham Pharmacia Biotech Toronto, ON, Canada) following the manufacturer’s procedure. Then cDNA was acted as a sample plate for polymerase chain reaction (PCR) extension together with SYBR Green (Takara, Dalian, China). Real-time PCR was conducted by Thermal Cycler Dice Real-Time PCR System (Takara Bio, Shiga, Japan). The expression levels of target genes were figured by employing the $2^{-\text{ΔΔ}C_{\text{t}}}$ method, which were, respectively, standardized to glyceraldehyde 3-phosphate dehydrogenase (GAPDH) and U6. The primers used for qRT-PCR (Bioneer Technology, Alameda, CA, U.S.A.) were as follows.

NR2F2-AS1:5′-TCAGCCGGAAAACTACAAGCTC-3′ (forward),
NR2F2-AS1: 5′- TCTTCGTGTAGCTGTTCCACC -3′ (reverse);
miR-4429: 5′-GGCCAGGCAGTCTGAGTTG-3′ (forward),
miR-4429: 5′-GGGAGAAAAGCTGGGCTGAG-3′ (reverse);
MBD1: 5′-CTGCATCTGCGTCTTCACAT-3′ (forward),
MBD1: 5′-CACACCCCACAGTCCTCTTT-3′ (reverse);
GAPDH: 5′-GAAGGTGAAGGTCGGAGTC-3′ (forward),
GAPDH: 5′-GAAGATGGTGATGGGATTTC-3′ (reverse);
U6: 5′-GCTTCGGCAGCACATATACTAA AAT-3′ (forward),
U6: 5′-CGCTTCACGAATTTGCGTGTCAT-3′ (reverse).

### Western blot analysis

Proteins were extracted by using RIPA lysis buffer (Beyotime Biotechnology, China) supplemented with protease inhibitors (Roche, China). Afterwards, these proteins were quantified with the use of BCA™ Protein Assay Kit (Pierce, Appleton, U.S.A.). Cell proteins were separated by using 10% sodium dodecyl sulfate-polyacrylamide gel electrophoresis, and then transferred to the polyvinylidene difluoride (PVDF) membranes. The membrane was blocked in 5% skim milk and incubated with primary antibodies overnight at 4°C, followed by cultivation with secondary antibodies for over 2 h at room temperature. Protein bands were detected by the ECL chemiluminescent Detection System (Thermo Fisher Scientific, Rochester, NY, U.S.A.). The primary antibodies were list as follows: E-cadherin (ab1416, Abcam, U.K.), N-cadherin (ab18203, Abcam), MBD1 (ab2846, Abcam), GAPDH (ab8245, Abcam). GAPDH served as the internal control.

### Cell proliferation assay

Cell Counting Kit-8 (CCK-8; Dojindo Molecular Technologies, Inc., Kyushu, Japan) was used to study cell proliferation. Cell proliferation was probed at 0, 24, 48, and 72 post transfection. In brief, 10 μl of CCK-8 reagent was added to each well, cells then were incubated at 37°C. After 4 h, cell proliferation was found at a wavelength of 450 nm by the microplate reader (EL340; BioTek Instruments, Hopkinton, MA, U.S.A.). Assays were carried out three times independently.

### Colony formation assay

Transfected cells were plated on 6-well plates at the density of 1000 cells per well. Then transfected cells were cultured in DMEM involving 10% FBS and replaced the medium every 3 days. Afterward, cells were cultured for 2 weeks in a humid incubator with 5% CO_2_ at 37°C. The cells were fixed by using methanol and stained by crystal violet. The colony numbers then were counted manually.

### Flow cytometry analysis

In brief, transfected cells were collected and resuspended with phosphate-buffered saline (PBS). Transfected cells were double stained by propidium iodide and Annexin V-fluorescein isothiocyanate in accordance with manufacturer’s instruction. In the end, cell apoptosis was demonstrated by using flow cytometry (BD Biosciences, Franklin Lakes, NJ, U.S.A.).

### Transwell assay

Transfected cells were added on upper chambers which were coated with Matrigel and contained serum-free DMEM (Gibco, Waltham, MA, U.S.A.). DMEM containing 10% FBS was added to the lower chamber. Transfected cells were cultured for 48 h in a humid incubator at 37°C with 5% CO_2_. Noninvasive cells were cleared by a cotton swab, and the invaded cells were fixed with the application of methanol and stained with crystal violet. The number of invaded cells was counted under a light microscope (Olympus Corporation, Tokyo, Japan). Cell migration was studied as invasion assays except the upper chambers without Matrigel. The experiments were conducted in triplicate.

### Luciferase reporter assay

The pmirGLO-NR2F2-AS1-WT or pmirGLO-NR2F2-AS1-Mut vectors were co-transfected, respectively, with NC mimics or miR-4429 mimics vectors into cells. pmirGLO-MBD1-WT or pmirGLO-MBD1-Mut vectors were co-transfected with NC mimics or miR-4429 mimics vectors respectively into cells. Lipofectamine 2000 was used for transfection. After 48 h, the relative luciferase activities were detected by using luciferase reporter assay system (Promega, Madison WI, U.S.A.).

### RNA pull-down assay

Pull-down assay was utilized to examine the underlying binding capacity between NR2F2-AS1 with miR-4429. NR2F2-AS1-Wt, NR2F2-AS1-Mut, and NC were biotinylated to be Bio-NR2F2-AS1-Wt, Bio-NR2F2-AS1-Mut, and Bio-NC by GenePharma Company (Shanghai, China). Bio-NR2F2-AS1-Mt, Bio-NR2F2-AS1-Mut and Bio-NC were transfected into HeLa or SiHa cells. After incubation of 48 h, cells were lysed, and the cell lysate was cultured with Dynabeads M-280 Streptavidin (Invitrogen, CA). Purified RNA complex was detected by qRT-PCR.

### RIP assay

RIP assay was conducted by utilizing Magna RNA-binding protein immunoprecipitation kit (Millipore, Billerica, MA, U.S.A.). Magnetic beads coated with human anti-Ago2 antibody were added to the mixture of RIP buffer and cell lysate. Normal IgG was regard as negative control. Then, proteinase K was used to purify RNA. Purified RNAs were utilized to quantitative real-time PCR (qRT-PCR).

### Statistical analysis

SPSS 20.0 Software (SPSS Inc., Chicago, IL, U.S.A.) was used for data analysis. Student’s *t-*test and One-way analysis of variance were utilized to analyze differences of each group. Associations among target genes were analyzed with Spearman’s correlation analysis. Data were shown as the mean ± SD. All experiments were repeated three times. *P*<0.05 was considered significant.

## Results

### NR2F2-AS1 expression is up-regulated in cervical cancer tissues and cells

To investigate the potential role of NR2F2-AS1 in cervical cancer, we detected the relative expression of NR2F2-AS1 in cervical cancer tissues and cells. Our study found that NR2F2-AS1 was significantly up-regulated in cervical cancer tissues compared with matched healthy tissues (Figure 1A). NR2F2-AS1 expression was prominently increased in cervical cancer cell lines (HeLa, SiHa, C33A, and C4-1) in comparison with the normal human cervical cells (Ect1/E6E7) (Figure 1B). Furthermore, we observed the increased expression of NR2F2-AS1 in advanced stages of patients with cervical cancer (Figure 1C). In conclusion, the results above reveal that NR2F2-AS1 is highly expressed in cervical cancer tissues and cell lines, especially in patients with advanced cervical cancer.

**Figure 1:** NR2F2-AS1 is up-regulated in cervical cancer tissues and cell lines and contributes to poor prognosis of patients (**A**) qRT-PCR assay was conducted to assess NR2F2-AS1 expression in cervical cancer tissues and matched adjacent tissues. (**B**) qRT-PCR assay detected that expression level of NR2F2-AS1 in cervical cancer cell lines (HeLa, SiHa, C33A, and C4-1) and in normal human cervical cells (Ect1/E6E7). (**C**) qRT-PCR assay was conducted to detect NR2F2-AS1 expression in different clinical stages. *P<0.05, **P<0.01 versus control group.

### Down-regulation of NR2F2-AS1 inhibits proliferation, migration, invasion in cervical cancer cells

Based on the investigations above, the effects of NR2F2-AS1 down-regulation on cell proliferation, migration, invasion were detected in HeLa and SiHa cells. We discovered that NR2F2-AS1 knockdown inhibited proliferation ability and colony formation, whereas facilitated cell apoptosis in HeLa and SiHa cells (Figure 2A–C). Furthermore, the transwell assay demonstrated that knockdown of NR2F2-AS1 hampered the migration and invasion of HeLa and SiHa cells (Figure 2D,E). Because epithelial-mesenchymal transition (EMT) plays a critical role in cancer cell migration and invasion, we conducted Western blot assay to confirm whether NR2F2-AS1 had effect on the process of EMT in cervical cancer. Our results showed that the expression of the epithelial marker E-cadherin was prominently up-regulated, and the mesenchymal marker N-cadherin expression was dramatically reduced by silenced NR2F2-AS1 in cervical cancer (Figure 2F). In a word, NR2F2-AS1 knockdown inhibits proliferation, migration and invasion in cervical cancer cells.

**Figure 2:** NR2F2-AS1 knockdown suppresses the malignant behaviors of cervical cancer cells (**A,B**) The CCK8 and colony formation assays were conducted to investigate cell proliferation. (**C**) Flow cytometry analysis was carried out to explore cell apoptosis rate. (**D,E**) Cell migration and invasion were probed by transwell assays. (**F**) The expression of EMT-relevant proteins were researched by Western blot analysis. *P<0.05 control group.

### NR2F2-AS1 acts as a sponge of miR-4429 in cervical cancer

Since accumulating studies exhibit that lncRNAs could function as competing endogenous RNAs (ceRNAs) to sponge miRNAs in cancers [15,16], we intended to investigate whether NR2F2-AS1 could interact with miRNAs in cervical cancer. We searched starBase database and found seven miRNA that can bind with NR2F2-AS1 (strict stringency (≥5)). RNA pull down showed that miR-4429 had the most significant effect (Figure 3A). It was confirmed that the expression of miR-4429 was obviously declined in cervical cancer cells compared with normal cervical cells (Figure 3B). Next, we verified miR-4429 mimics vector led to dramatical rise of miR-4429 expression (Figure 3C). The binding sites between miR-4429 and NR2F2-AS1 were found from starBase (Figure 3D). To confirm the interaction between NR2F2-AS1 and miR-4429, we carried out luciferase assay. The result suggested that luciferase activity of pmirGLO-NR2F2-AS1-Wt was obviously decreased in miR-4429 mimics transfected cells, while pmirGLO-NR2F2-AS1-Mut showed no significant change between miR-4429 mimics group and miR-NC group (Figure 3E). RIP assay indicated that NR2F2-AS1 and miR-4429 were enriched in Ago2 groups but not in IgG groups (Figure 3F). Additionally, to further investigate the interaction between NR2F2-AS1 and miR-4429, we carried out the qRT-PCR experiments and confirmed that miR-4429 overexpression led to a significant reduction of NR2F2-AS1 (Figure 3G). Moreover, Spearman’s correlation analysis verified the negative correlation between NR2F2-AS1 and miR-4429 (Figure 3H). Therefore, we draw a conclusion that miR-4429 is sponged by NR2F2-AS1 in cervical cancer.

**Figure 3:** NR2F2-AS1 acts as a sponge for miR-4429 in cervical carcinoma (**A**) StarBase v2.0 database detected the miRNAs that can bind with NR2F2-AS1, and RNA pull-down assay assessed the expression level of miR-4429 comparing with the other miRNAs. (**B**) qRT-PCR assay was conducted to evaluate miR-4429 expression in cervical cancer cells and normal cervical cells. (**C**) The effects of miR-4429 mimics were proved by qRT-PCR assay. (**D**) The underlying binding sites between miR-4429 and NR2F2-AS1 were speculated by starBase v2.0 database. (**E,F**) Luciferase reporter and RIP assays were performed to verify the interaction between miR-4429 and NR2F2-AS1. (**G**) The expression of NR2F2-AS1 in miR-4429 mimics-treated cervical cancer cells was detected through qRT-PCR assay. (**H**) The correlation of miR-4429 and NR2F2-AS1 was probed by Spearman's correlation analysis. *P<0.05 versus control group.

### MBD1 is the downstream target of miR-4429

Then the target gene of miR-4429 in cervical cancer was explored, we found nine candidate genes that could bind with miR-4429 by starBase v2.0 software (Figure 4A). Then, we found that miR-4429 overexpression contributed to the most distinct reduction of MBD1 in comparison with the other candidate genes (Figure 4B). It was verified that the expression of MBD1 was prominently increased in cervical cancer cells compared with normal cervical cells (Figure 4C). Bioinformatics confirmed the 3′-UTR of MBD1 included the binding site of miR-4429 (Figure 4D). Hence, MBD1 was chosen for the further study. Luciferase assay demonstrated that luciferase activity of pmirGLO-MBD1-Wt was obviously decreased by the introduction of miR-4429 mimics vector, but no distinct change was detected in pmirGLO-MBD1-Mut groups (Figure 4D). RIP assay revealed that MBD1 and miR-4429 were enriched in Ago2 groups but not in IgG groups, suggesting that MBD1 was the downstream target of miR-4429 (Figure 4E). Furthermore, we found that the mRNA and protein expression of MBD1 were declined by miR-4429 mimics transfected cervical cancer cells in qRT-PCR and Western blot (Figure 4F). To sum up, MBD1 is a downstream target of miR-4429.

**Figure 4:** MiR-4429 targets MBD1 and is negatively correlated to MBD1 expression (**A,B**) Nine candidate genes that could bind with miR-4429 were assessed by starBase v2.0 software, and qRT-PCR assay proved that MBD1 had the most obvious effect. (**C**) qRT-PCR assay showed the expression level of MBD1 in cervical cancer cells. (**D,E**) The interaction between miR-4429 and MBD1 was confirmed by luciferase reporter assay and RIP assay. (**F**) The mRNA and protein expression of MBD1 were proved by qRT-PCR and Western blot assay. *P<0.05 versus control group.

### NR2F2-AS1 promotes cervical cancer progression via regulating MBD1

Finally, we demonstrated whether NR2F2-AS1 promoted the progression of cervical cancer by targeting miR-4429/MBD1 axis. We found that the introduction of pcDNA3.1/MBD1 vector could lead to prominent rise of MBD1 expression (Figure 5A). As shown in Figure 5B–D, MBD1 up-regulation reversed the inhibitory effects of NR2F2-AS1 knockdown on the proliferation, colony formation of cervical cancer cells, but counteracted the elevated percentage of apoptotic cells resulted from NR2F2-AS1 knockdown. Western blot assay revealed that MBD1 up-regulation counteracted the NR2F2-AS1 knockdown-mediated inhibition on EMT progression. Furthermore, suppression of NR2F2-AS1 led to the decrease in MBD1 expression, and MBD1 overexpression recovered the expression of MBD1 suppressed by NR2F2-AS1 knockdown (Figure 5E). According to the results above, we draw a conclusion that NR2F2-AS1 promotes the progression of cervical cancer via targeting miR-4429/MBD1 axis.

**Figure 5:** NR2F2-AS1 accelerates cervical carcinoma progression through sponging miR-4429 to regulate MBD1 expression (**A**) The effect of MBD1 overexpression was detected by qRT-PCR assay. (**B,C**) Cell proliferative ability was determined by CCK8 and colony formation assays. (**D**) Flow cytometry was performed to evaluate cell apoptosis. (**E**) Western blot assay was conducted to assess the EMT process. *P<0.05 versus control group.

## Discussion

Accumulating literature has unveiled that NR2F2-AS1 is an oncogene in some cancers, including prostate carcinoma, non-small cell lung cancer, and colorectal cancer [12–14]. However, the biological role and corresponding regulatory mechanism of NR2F2-AS1 in cervical cancer remain unclear. The present study disclosed that NR2F2-AS1 expression was dramatically up-regulated in cervical cancer tissues and cells, and high NR2F2-AS1 expression was linked to poor prognosis of cervical cancer patients. Moreover, knockdown of NR2F2-AS1 greatly inhibited the progression of cervical cancer by impeding cell proliferation, migration, invasion, and EMT as well as promoting cell apoptosis.

Then, we aimed to investigate the potential mechanism of NR2F2-AS1 regulating cervical cancer development. LncRNAs are likely to serve as a molecule sponge for microRNAs (miRNAs) in the regulation of cancers [17]. For example, lncRNA LUCAT1 fosters cell proliferation and invasion in gastric cancer through targeting miR-134-5p [18]. LncRNA HOTAIR increases the expression of HER2 via sponging miR-331-3p to drive gastric cancer growth and invasion [19]. LncRNA CCAT1 facilitates cell proliferation, migration and invasion by competing for miR-143 in thyroid carcinoma [20]. Unlike lncRNAs, miRNAs are short non-coding RNAs of approximately 22 nucleotides [21]. Increasing researches have confirmed the functions of miRNAs in cancers. For instance, miR-10a is highly expressed in non-small cell lung cancer and may exacerbate cancer by down-regulating PTEN [22]. MiR-27a enhances ovarian cancer development via repressing FOXO1 [23]. MiR-30 family members suppress breast cancer invasion through targeting multiple bone metastasis-related genes [24]. And in this paper, we predicted the combination of NR2F2-AS1 and miR-4429. Of note, miR-4429 functions as a tumor inhibitor in some cancers. For example, miR-4429 obstructs gastric cancer progression by binding with METTL3 [25]. MiR-4429 promotes cervical cancer cell radio-sensitivity through RAD51 [26]. MiR-4429 suppresses cell proliferation, migration, invasion, and EMT via modulating CDK6 in clear cell renal cell carcinoma [27]. Furthermore, miR-4429 was proved to be sponged and negatively regulated by NR2F2-AS1 in cervical cancer.

It has been demonstrated that miRNAs can bind with target messenger RNAs (mRNAs) to affect cancer biology [28]. MBD1 was hereby speculated as the target gene of miR-4429 in cervical cancer. As an oncogene, MBD1 promotes cell proliferation and metastasis in gallbladder cancer [29]. MBD1 inhibition obstructs pancreatic cancer cell invasion and EMT via E-cadherin down-regulation [30]. MBD1 increases pancreatic cancer therapy resistance through DNA repair [31]. Further, our study confirmed that MBD1 interacted with miR-4429 cervical cancer and NR2F2-AS1 up-regulated MBD1 by competing for miR-4429 in cervical cancer. In the end, rescue assays unveiled that NR2F2-AS1 enhanced the development of cervical cancer through miR-4429/MBD1 axis.

In summary, our work firstly illuminated that NR2F2-AS1 contributed to the development of cervical cancer via sponging miR-4429 to regulate MBD1, which may be beneficial to cervical cancer treatment in the future.

## Abbreviations

ATCC: American Type Culture Collection
CCK‐8: Cell Counting Kit‐8
cDNA: complementary DNA
DMEM: Dulbecco’s modified Eagle’s medium
EMT: epithelial-mesenchymal transition
FBS: fetal bovine serum
GAPDH: glyceraldehyde 3-phosphate dehydrogenase
lncRNAs: long noncoding RNAs
MBD1: methyl-CpG-binding domain protein 1
miRNAs: microRNAs
mRNAs: messenger RNAs
NR2F2-AS1: NR2F2 antisense RNA 1
PVDF: polyvinylidene difluoride
qRT‐PCR: quantitative real-time PCR
